# Identification of RegIV as a Novel GLI1 Target Gene in Human Pancreatic Cancer

**DOI:** 10.1371/journal.pone.0018434

**Published:** 2011-04-11

**Authors:** Feng Wang, Ling Xu, Chuanyong Guo, Aiwu Ke, Guoyong Hu, Xuanfu Xu, Wenhui Mo, Lijuan Yang, Yinshi Huang, Shanshan He, Xingpeng Wang

**Affiliations:** 1 Department of Gastroenterology, The First People's Hospital, Shanghai Jiao Tong University School of Medicine, Shanghai, People's Republic of China; 2 Department of Gastroenterology, The Tenth People's Hospital of Shanghai, Tongji University, Shanghai, People's Republic of China; University of South Florida College of Medicine, United States of America

## Abstract

**Background and Aims:**

GLI1 is the key transcriptional factor in the Hedgehog signaling pathway in pancreatic cancer. RegIV is associated with regeneration, and cell growth, survival, adhesion and resistance to apoptosis. We aimed to study RegIV expression in pancreatic cancer and its relationship to GLI1.

**Methods:**

GLI1 and RegIV expression were evaluated in tumor tissue and adjacent normal tissues of pancreatic cancer patients and 5 pancreatic cancer cell lines by qRT-PCR, Western blot, and immunohistochemistry (IHC), and the correlation between them. The GLI1-shRNA lentiviral vector was constructed and transfected into PANC-1, and lentiviral vector containing the GLI1 expression sequence was constructed and transfected into BxPC-3. GLI1 and RegIV expression were evaluated by qRT-PCR and Western blot. Finally we demonstrated RegIV to be the target of GLI1 by chromatin immunoprecipitation (CHIP) and electrophoretic mobility shift assays (EMSA).

**Results:**

The results of IHC and qRT-PCR showed that RegIV and GLI1 expression was higher in pancreatic cancer tissues versus adjacent normal tissues (p<0.001). RegIV expression correlated with GLI1 expression in these tissues (R = 0.795, p<0.0001). These results were verified for protein (R = 0.939, p = 0.018) and mRNA expression (R = 0.959, p = 0.011) in 5 pancreatic cancer cell lines. RegIV mRNA and protein expression was decreased (94.7±0.3%, 84.1±0.5%; respectively) when GLI1 was knocked down (82.1±3.2%, 76.7±2.2%; respectively) by the RNAi technique. GLI1 overexpression in mRNA and protein level (924.5±5.3%, 362.1±3.5%; respectively) induced RegIV overexpression (729.1±4.3%, 339.0±3.7%; respectively). Moreover, CHIP and EMSA assays showed GLI1 protein bound to RegIV promotor regions (GATCATCCA) in pancreatic cancer cells.

**Conclusion:**

GLI1 promotes RegIV transcription by binding to the RegIV gene promoter in pancreatic cancer.

## Introduction

Pancreatic cancer (PC) is the fourth most common cancer-related cause of mortality in the Western world [1]–[3] and has a dismal prognosis despite considerable progress in management. The median survival of PC is less than 6 months; the 5-year survival rate is less than 5% [1], [2]. More than 80% present with unresectable disease; one-third have local disease while the remainder have distant metastases. Research over the last two decades has shown that PC is a genetic disease fundamentally, caused by inherited germline and acquired somatic mutations in cancer-associated genes. Tumor progression model for PC in which the pancreatic ductal epithelium progresses from normal to increased grades of pancreatic intraepithelial neoplasia (PanINs) to invasive cancer. Multiple alterations in genes that are important in PC progression have been identified, for example K-ras, INK4A, p53, and SMAD4/DPC4 [4], [5]. PC is characterized by near-universal mutations in K-ras and frequent deregulation of crucial embryonic signalling pathways, including the Hedgehog (HH) signaling pathway [6], [7]. A better understanding of the mechanisms underlying the development of PC might help to improve early diagnosis and potentially identify molecular therapeutic targets.

The hedgehog (HH) signaling pathway was first identified in the embryonic development of Drosophila [8] and has been shown to be crucial for growth and patterning in the pancreas during embryonic development. HH signaling regulates cell differentiation and organ formation during embryonic development , and is expressed in pancreatic epithelial cells [9], [10]. Constitutive activation of HH signaling is detected in a variety of human cancers, including pancreatic cancer [9]–[13]. Given its misexpression in both metastatic pancreatic cancer cell lines and in precursor lesions (PanIN) [14], HH signal activation may be involved in both early and late pancreatic tumorigenesis.

Of the three mammalian ligands in the HH family, Sonic (SHH), Desert (DHH), and Indian (IHH) Hedgehog [15], the former has been associated with both pancreatic organogenesis and pancreatic cancer. HH signals are transmitted and modified by two transmembrane proteins, patched (PTCH) and smoothened (SMO), and by downstream transcription factors that are members of the glioma-associated oncogene (GLI) family (GLI1, 2, and 3). GLI2 and GLI3 have transactivation and repressive domains, whereas GLI1 likely functions only as a transactivator and transcriptional target of the HH pathway itself [16]–[19]. The regenerating gene (Reg) family, a group of small secretory proteins, is involved in cell proliferation or differentiation in digestive organs [20], is upregulated in several gastrointestinal cancers, and functions as trophic or antiapoptotic factors [21]–[23]. RegIV, a member of the regenerating gene family, is involved in digestive tract malignancies, including the stomach [24], colorectum [25], [26], and pancreas [27], [28], as well as in benign diseases such as ulcerative colitis [29]. RegIV overexpression in tumor cells has been associated with cell growth, survival, adhesion, and resistance to apoptosis. Recently, RegIV overexpression was reported to be associated with the initiation and progression of pancreatic cancer, and was suggested as a promising tumor marker to screen early stage PC and target for adjuvant therapy in PC [28], [30].

The functions of GLI1 and RegIV appeared to be similar in our review of the literature; thus, we investigated the expression and correlation of GLI1 and RegIV in PC tissues and cell lines. We also explored the possible mechanism between GLI1 and RegIV, by using ChIP and EMSA assays.

## Materials and Methods

### Cell lines and tissues

Human pancreatic cancer cell lines, PANC-1, AsPC-1, BxPC-3, CaPan-2 and SW1990, were purchased from Chinese Academy of Sciences Committee Type Culture Collection cell bank. PANC-1 was cultured in Dulbecco's Modified Eagle's Medium (DMEM) (Gibco BRL, USA), the other types of Cells were cultured in RPMI-1640 (Gibco BRL, USA), and all the mediums were supplemented with 10% FBS (Gibco BRL, USA), penicillin G (100 U/ml), streptomycin (100 ug/ml). Cells were incubated at 37°C with 5% CO2. Twelve pairs of PC and corresponding non-cancerous pancreas tissues were obtained from Shanghai Tenth People's Hospital with full written ethical consent. None of these patients had received chemotherapy or radiation therapy prior to cancer resection. Another 9 paired tissues slices was obtained from pathology department of Shanghai Tenth People's Hospital. The study was approved by the Ethical Committee of Tongji University School of Medicine and Life Sciences.

### Short Hairpin RNA (shRNA) Design and Vector Production

Interfering sequences corresponding to distinct regions of GLI1mRNA, as well as negative control with no homology for human or mouse genes were designed by Shanghai GeneChem Biotech (Table 1). Three siRNA duplexes were screened for GLI1 knock-down by Western blot analysis in cotransfection experiments with GLI1 expression plasmid in HEK 293T cells. The most successful sequence and one non-silencing Luciferase sequence were designed into a shRNA oligonucleotide template consisting of sense, hairpin loop, antisense, and terminator sequences, all of which were flanked by restriction enzyme sites to facilitate directional sub-cloning. The resulting vectors encoded GFP under transcriptional control of the EF1 promoter and a H1 promoter upstream of cloning restriction sites (*Mlu*I and *Cla*I) to allow the introduction of oligonucleotides encoding shRNAs. Either shRNA against GLI1 or a nonsilencing-Luciferase shRNA was located under the H1 promoter (Figure 1). The correct insertion of the specific shRNA was further confirmed by direct DNA sequencing.

**Figure 1:** Construction of the pLVTHM vector encoding anti-GLI1 shRNA. For the GLI1-shRNA vector, two single strand DNAs encoding two linkers, the target sequences and a loop element, were synthesized. These were annealed to double stranded DNA, and ligated into the pLVTHM following *Mlu*I and *Cal*I digestion. The short hairpin form of shGLI1 is expressed under the control of human H1 promoter. The vector also contains a human EF1-α promoter driving the GFP marker gene for tracking transduced cells. The vectors were generated by transient transfection of pRsv-REV, pMDlg-pRRE, pMD2G, and the shRNA encoding pLVTHM into 293T cells. Abbreviations: RRE, Rev response element; cPPT, central polypurine tract; EF1-α, human elongation factor 1-α promoter; H1, the human H1 promoter; GFP, green fluorescent protein; PRE, human hepatitis virus posttranscriptional regulatory element.

**Table 1:** Sequences of primers used in this study for GLI1-shRNA constructs.

5'		STEMP	Loop	STEMP
shGLI1-1	CGCGTCCCC	CTCCACAGGCATACAGGAT	TTCAAGAGA	ATCCTGTATGCCTGTGGAG
	CGATTTCCAAAAA	CTCCACAGGCATACAGGAT	TCTCTTGAA	ATCCTGTATGCCTGTGGAG
shGLI1-2	CGCGTCCCC	CGTGAGCCTGAATCTGTGTAT	TTCAAGAGA	ATACACAGATTCAGGCTCACG
	CGATTTCCAAAAA	CGTGAGCCTGAATCTGTGTAT	TCTCTTGAA	ATACACAGATTCAGGCTCACG
shGLI1-3	CGCGTCCCC	GCTCAGCTTGTGTGTAATTAT	TTCAAGAGA	ATAATTACACACAAGCTGAGC
	CGATTTCCAAAAA	GCTCAGCTTGTGTGTAATTAT	TCTCTTGAA	ATAATTACACACAAGCTGAGC
scramble	CGCGTCCCC	GCCAGCGTTAACCAGACTA	TTCAAGAGA	TAGTCTGGTTAACGCTGGC
	CGATTTCCAAAAA	GCCAGCGTTAACCAGACTA	TCTCTTGAA	TAGTCTGGTTAACGCTGGC

For production of the lentiviral vector, HEK 293T cells were cultured to 30–40% confluence by the following day. The next day, the medium was replaced with DMEM/10% FBS without antibiotics. Subsequently, 20 µg of shRNA plasmid DNA (nonsense shRNA or GLI1 targeting shRNA; GeneChem Biotech, Shanghai, China), 7.5 µg pMD2G, 10 µg pRsv-Rev, and 15 µg pMDLg-pRRE were mixed with sterile ddH_2_O to a final volume of 1800 µl, then mixed with 200 µl of 2.5 M CaCl_2_. The DNA mix was oxygenated and 2000 µl 2×PBS (pH 7.05) added in drops, and incubated at room temperature for 30 minutes. The transfection mixture was added to its respective plates and incubated overnight. The medium was replaced after 12 hours with DMEM supplemented with 10% FBS. After 48 hours, the conditioned medium containing shRNA lentivirus was collected and filtered through 0.45-µm pore size cellulose acetate filters, and stored on ice. The virus was concentrated by spinning at 70,000 G for 2 hours and resuspended with 500 µl PBS. The transduction unit (TU) titer was assessed on HEK 293T cells in the presence of polybrene 8 µg/mL (Sigma-Aldrich, St. Louis, MO, USA). Titers of 2–5×10^8^ TU/ml were routinely achieved.

### Overexpression-GLI1 Lentiviral Vector Construction

Human GLI1 cDNA was purchased from Open-Biosystem (USA). The complete cDNA sequence of GLI1 was generated by PCR using the forward primer, 5′-GAGGATCCCCGGGTACCGGTCGCCACCATGTTCAACTCGATGACCCCAC-3′; and reverse primer, 5′-TCATCCTTGTAGTCGCTAGCGGCACTAGAGTTGAGGA-3′; then inserted into a pGC-FU-EGFP-3FLAG Vector (GeneChem Company, Shanghai, China). Transformants were analyzed by sequencing. The resultant 3320-bp fragment was confirmed by sequencing (Figure S1) and compared with the sequence of the GLI1 gene expression region in GenBank (NM_005269.2). To produce lentiviral stock, 293FT cells were cultured to 70–85% confluence the following day. The complete culture medium was removed. Cells were then exposed to 5 mL medium (Opti-MEM; Invitrogen) with complexes containing packaging helper construct (GeneChem Company, Shanghai, China), 20 µg expression plasmid DNA (pGC-FU-EGFP-3FLAG-GLI1), or control plasmid DNA (pGC-FU-EGFP-3FLAG) with 100 µl lipofectamine 2000 (Invitrogen, USA) in the presence of polybrene (8 µg/mL, Sigma-Aldrich, St. Louis, MO, USA). After incubation for 24 hours, the infection medium was replaced with complete culture medium. Lentivirus-containing supernatants were harvested 72 hours after transfection. The supernatants were centrifuged to remove pellet debris and stored at −80°C. Titers of 2–5×10^7^ TU/ml were routinely achieved.

### Lentiviral Transfection

Cells (1×10^5^) in a six-well plate were transfected with the lentiviral vector at a multiplicity of infection (MOI) = 5 (PANC-1) or 20 (BxPC-3) in the presence of 8 µg/ml polybrene (Sigma-Aldrich, St. Louis, MO, USA). After 72 hours of transfection, the medium was replaced with 2 ml complete culture medium. 48 hours after transfection, GLI1 expression was established by real time-PCR and Western blot analysis.

### Flow Cytometry

Cells were adjusted to 1×10^6^ cells/100 µL and used for flow cytometry. A total of 10,000 events were analyzed to determine transfection efficiency using FACS Calibur (Becton Dickinson, USA) Cell-Quest software.

### qRT-PCR

Real-time quantitative reverse-transcription polymerase chain reaction (qRT-PCR) analysis was performed with the ABI Prism 7900HT Sequence Detection System (Applied Biosystems, CA, USA). GLI1 and RegIV mRNA expression was analyzed by qRT-PCR using SYBR Green Dye. β-actin was used as the housekeeping gene. Target gene expression was normalized to β-actin and analyzed by the 2*^−ΔΔCT^* formula. The primer sequences are as follows: GLI1, forward: TTCCTACCAGAGTCCCAAGT, reverse: CCCTATGTGAAGCCCTATTT, RegIV, forward: CGCTGAGATGAACCCCAAG, reverse: TGAGAGGGAAGTGGGAAGAG. β-actin, forward: AAGGGACTTCCTGTAACAATGCA, reverse: CTGGAACGGTGAAGGTGACA. All reactions were performed at least three times.

### Western blot analysis

Cells were rinsed twice in PBS, then lysed for 2 hours in RIPA lysis buffer on ice and centrifuged at 12,000 rpm for 10 minutes at 4°C. Protein concentration was determined by the standard BCA method (BCA™ Protein Assay Kit, Pierce, USA). 50 µg of total protein was separated by SDS-PAGE using 6% or 12% polyacrylamide gel with Mini-PROTEAN Tetra Cell (Bio-Rad, USA). GLI1 and RegIV protein in gel was transferred to a 0.45-µm nitrocellulose membrane with Mini Transfer Cell and Trans-blot SD Semi-Dry Transfer Cell (Bio-Rad, USA) respectively.

The immunoreagents used for Western blot were rabbit monoclonal antibody against GLI1 (1∶200; Santa Cruz, USA) and goat polyclonal anti-RegIV antibody (1∶100; Santa Cruz, USA). Mouse polyclonal anti-β-actin antibody (1∶5000; Santa Cruz, USA) was used as loading control. The blots were developed by a standard enhanced chemiluminescence (ECL) method (Pierce, USA). All experiments were repeated several times and gave similar results.

### Immunohistochemistry

Tumor sections were deparaffinized, rehydrated, and treated with 10 mM citrate buffer (pH 6.0) at 95°C to retrieve antigens. After quenching endogenous peroxidase activity with H_2_O_2_ and blocking with 10% normal horse serum, the sections were incubated sequentially with the primary antibodies goat anti-RegIV (1∶100; Santa Cruz, California, USA), rabbit anti-GLI1 (1∶200; Santa Cruz, California, USA), biotinylated secondary antibodies, and the ABC reagent (Gene Tech, Shanghai, China). The immunostaining was visualized with 3.3-diaminobenzidine (Gene Tech, Shanghai, China). The sections were then counterstained with hematoxylin. Negative controls were performed in each case by replacing the primary antibody with PBS.

### Chromatin immunoprecipitation (CHIP)

We modified the previously reported protocol [31] for chromatin immunoprecipitation (CHIP). In brief, PANC-1 cells (3×10^7^) were cross-linked with 1% formaldehyde. The fixation reaction was stopped by adding 10 ml Glycin (0.125 M), then chromatin was collected with 1 mL IP buffer containing protease inhibitor cocktails. Chromatin was sheared by using a sonicator with a 4 mm tip probe 3 times for 10 second pulses (60 W, 80 W, and 100 W, respectively, 90 s intervals) in an ice box. Crosslinking was reversed by adding 20 µL of 5 M NaCl overnight at 65°C. DNA was extracted using phenol/chloroform assay. 20 µL of DNA was electrophoresed on a 1.5% agarose gel and the rest was preserved at −20°C as INPUT DNA. Soluble chromatin was immunoprecipitated with 2 µg anti-GLI1 rabbit monoclonal antibody (Santa Cruz, California, USA). The 2 µg mouse IgG (Santa Cruz, California, USA) was added as a random control, RNA polymerase II as a positive control, and β-actin antibody as a negative control. DNA-protein immune complexes were eluted and reverse cross-linked, and DNA was extracted with phenol/chloroform and precipitated. The presence of the RegIV promoter domain containing GLI1 motifs in immunoprecipitated DNA was identified by PCR using the following primers: RegIV-A for site 1 (118 bp), forward: 5′-5-TGGTCCCTTCCAGACTTA-3-3′, reverse: 5′- TCCAGTATAGATGGCAAA -3′. RegIV-B for site 2 (131 bp), forward: 5′-CTAACCCTTTGCCATCTA -3′, reverse: 5′-GACCTGGACACTGAACCTTG-3′. RegIV-C for site 3 (70 bp), forward: 5′-CTATGCTGCTCACAAGGA-3′, reverse: 5′-GTGTTACATAACGGGTTT-3′. RegIV-D for site4 (70 bp), forward: 5′-TGTAACACACTCTGTTGATGTAAGC-3′, reverse: 5′- CTATTTGAGCTTCTCCCGCAG-3′. RegIV-E for sites 3 and 4 (226 bp), forward: 5′-CTCGGAAGGTTTCTAATC-3′, reverse: 5′- TTCAACATGCGTGAGTTT-3′. RegIV-F for sites 3 and 4 (481 bp), forward: 5′-CTATGCTGCTCACAAGGA-3′, reverse: 5′-AGACGGCTTCAGAATGTA-3′. RegIV-G for site 5 (315 bp), forward: 5′-TTCCTGAGGCAAGAAGAT-3′, reverse: 5′-CCAAGATTTAACCCAACA-3′. The PCR conditions for the RegIV promoter region were: denaturation 30 seconds at 94°C, annealing 30 s, elongation 1 minute at 72°C. Annealing temperatures for RegIV-A-G were 55°C, 56°C, 56°C, 47°C, 56°C, 56°C, and 52°C, respectively. The amplification of the RegIV promoter region was analyzed after 35 cycles. All experiments were repeated at least three times.

### Electrophoretic Mobility Shift Assays (EMSA)

Nuclear extracts were prepared with NE-PER Nuclear and Cytoplasmic Extraction Reagents (Pierce, Rockford, USA). EMSA and supershift EMSA with digoxin-labeled probes were performed using the DIG-Gel shift kit according to the manufacturer's instructions (Roche, Basel, Switzerland). The sequences of the oligonucleotides used were 5′-AGAACATGGATGATCATGTCA-3′ (binding motif underlined). Mutant oligonucleotides used were 5′-AGAACAAAAAATTTTATGTCA-3′. In the supershift study, 5 µg rabbit monoclonal antibody against GLI1 was incubated with 5 µg of nuclear extract on ice for 30 minutes before addition of the labeled probe, and further incubated on ice for 30 minutes. The entire 20 µl binding reaction was resolved on a 7% polyacrylamide gel and transferred to a positively charged nylon membrane (Bio-Rad, USA) in 0.5× Tris borate-EDTA buffer.

### Statistical analysis

Quantitative data are expressed as the mean ± standard deviation (SD). Real-time PCR data was analyzed according to the differences of target gene expression by the paired t-test and were 2*^−ΔΔCT^* transformed before analysis. The relationship between GLI1 and RegIV expression was analyzed using Spearman. IHC data was analyzed using the Chi-squared test. A p-value of less than 0.05 was considered statistically significant.

## Results

### GLI1 and RegIV expression in pancreatic cancer tissues

To study GLI1 and RegIV expression in PC, qRT-PCR and IHC were used in 12 paired biopsy tissues. GLI1 expression was higher in 9 cases (9/12) compared with adjacent normal pancreatic tissues (p = 0.011; Figure 2); RegIV expression was higher in 9 cases (9/12) (p = 0.011; Figure 2). There was a positive correlation between GLI1 and RegIV in PC tissues (R = 0.795, p<0.0001; Figure 2). On IHC, we found RegIV to be expressed only in beta cells of normal endocrine pancreatic tissues, which confirmed Oue's report [37]. On IHC, GLI1 and RegIV expression were higher in most PC compared with normal tissues (15/21 versus 4/21, p = 0.001; 14/21 versus 5/21, p = 0.005; respectively; Figure 3). 15 of 21 PC cases had high expression of GLI1 protein, among which 11 cases expressed high levels of RegIV protein (p = 0.001; Figure 3).

**Figure 2:** GLI1 and RegIV mRNA expression in PC tissues and adjacent normal tissues. The expression of GLI1 RegIV mRNA in 12 pairs of PC tissues and adjacent normal tissues(A–B). DNA from the samples were collected from surgical biopsies, and relative GLI1 and RegIV mRNA expression were detected by qRT-PCR. Statistical correlation between the expression of GLI1 and RegIV mRNA in 12 pairs of PC tissues and adjacent normal tissues was analyzed by Spearman's test (C). All results were normalized to β-actin mRNA expression. The data are presented as the mean ± SD and were calculated by the paired t-test. Significantly different between two groups: *p<0.05. ** p<0.01. NS: not significant.

**Figure 3:** Expression of GLI1 and RegIV proteins was analyzed by IHC in PC and adjacent normal tissues. All samples were collected, formalin-fixed, paraffin-embedded, and detected by IHC. Representative pictures are shown. Positive staining of GLI1 was observed at the PDAC cell nucleus (A); however, adjacent normal tissues exhibited no or faint staining for GLI1 (B). In adjacent normal pancreatic tissues, only islet cells showed positive staining of RegIV (D), while the positive staining of RegIV was observed as well as goblet-like cytoplasm granules in PC tissues (C). All photomicrographs were obtained at ×200 magnification. Scale bars, 100 µm.

### The correlation between GLI1 and RegIV

We tested GLI1 and RegIV expression in 5 PC cell lines by qPCR and Western blot. There was a positive correlation between the level of GLI1 and RegIV mRNA and protein (R = 0.958, p = 0.011 and R = 0.939, p = 0.018, respectively; Figure 4). GLI1 and RegIV were overexpressed in PC versus normal pancreatic cells.

**Figure 4:** The expression of GLI1 and RegIV in 5 PC cell lines. Expression of GLI1 and RegIV proteins in 5 pancreatic cancer cell lines as detected by Western blot analysis on cell extracts, using anti-GLI1 and anti-RegIV antibodies (A). β-actin was used as the loading control in all experiments. The results were quantified by determining the intensities of the bands compared with that of β-actin (B). Statistical correlation between expression of GLI1 and RegIV protein in 5 PC cell lines was analyzed by Pearson's test (C). Relative GLI1 and RegIV mRNA expression were examined by qRT-PCR (D). The expression of GLI1 and RegIV mRNA was normalized to β-actin mRNA expression. Statistical correlation between the expression of GLI1 and RegIV mRNA in 5 PC cell lines was analyzed by Pearson's test (E). All data are presented as the mean ± SD of three independent experiments.

### RegIV expression changed with GLI1 expression in PANC-1 and BxPC-3

To further verify the relationship between GLI1 and RegIV in PC cells, we designed and constructed shRNA-GLI1 lentiviral vector, and transfected it into PANC-1, a PC cell line with the highest expression of GLI1 (Figure 4). 48 hours after transfection, efficiency of transfection was shown by flow cytometry (FCM) to be more than 95% (Figure S2); stable fluorescence could still be detected even after 20 passages (Figure S3).

Afterwards, qRT-PCR and Western blot were used to detect RegIV expression in GLI1-shRNA-PANC-1 cells. Cells without transfection were used as controls, while cells transfected with scramble shRNA were used as negative controls. RegIV mRNA decreased by 94.7±0.3% when GLI1 mRNA decreased by 82.1±3.2%. RegIV protein decreased by 84.1±0.5% when GLI1 protein decreased by 76.7±2.2% (Figure 5). This suggested that RegIV expression decreased when GLI1 was silenced by RNAi.

**Figure 5:** RegIV expression changed with GLI1 in PC cells. PANC-1 cells were transfected with GLI1-shRNA or GFP-shRNA, BxPC-3 cells were transfected with LV-GLI1-eGFP or LV-eGFP, then expression of GLI1 mRNA relative to that of β-actin mRNA was assessed by qRT-PCR (A, D). After transfection, expression of GLI1 proteins was analyzed by Western blot (C, F). The inset shows a substantial decrease in RegIV expression by real-time RT-PCT (B, E) and Western blot analysis (C, F). The results were normalized to that of β-actin expression. All data are presented as the mean ± SD of three independent experiments.

We further designed and constructed a lentivirus vector that expressed GLI1, and transfected it into BxPC-3, with the lowest GLI1 expression in the 5 cell lines (Figure 4), to determine whether RegIV expression changed along with GLI1. 48 hours after transfection, qRT-PCR and Western blot were used to detect RegIV in the LV-GLI1-BxPC-3 cells. Cells without transfection were used as controls, while cells transfected with empty lentivirus vector were used as negative controls. RegIV mRNA increased by 729.1±4.3% when GLI1 mRNA increased by 924.5±5.3%. RegIV protein increased by 339.0±3.7% when GLI1 protein increased by 362.1±3.5% (Figure 5). This implies that RegIV expression increased when GLI1 was overexpressed. Based on these results, we concluded that GLI1, a transcription factor, might regulate RegIV gene expression.

### Identification of candidate Gli1 binding sites in the RegIV promoter

The positive correlation between GLI1 and RegIV in both PC tissue and cell lines prompted us to search the RegIV promoter for potential GLI1 binding sites to the DNA consensus sequence 5′-GACCACCCA-3′ [42]. Database analysis revealed four potential sites located upstream of the transcriptional start site (Figure 6). The homology of each GLI1 binding site to the canonical consensus sequence varied from 67% (sites 1, 2, 3, and 5) to 78% (site 4), which suggested that the RegIV gene promoter might bind to GLI1.

**Figure 6:** Potential GLI1 binding sites on the RegIV promoter and homology to the GLI1 consensus sequence. (A) Location of the potential GLI1 binding sites (numbers 1–5) in relation to the structure of the gene. P represents the transcriptional start site. The gray frame represents the variable splicing site. Blank frames represent exons. (B) Position of the binding sites on the promoter in relation to the P transcriptional start site and the sequence homology to the GLI1 consensus binding sequence, GACCACCCA.

### Confirmation of GLI1 protein bound to promoter region of RegIV gene by CHIP

The sonicated chromatin solution assay showed that the total DNA fragment appeared smeared in the 100 bp to 1 kb range in the 80 W group (Figure S4). The result of DNA electrophoresis showed the predicted DNA band in INPUT, GLI1-Ab, and postive control groups using human RegIV primer-D-F, and not in the IgG and negative control groups (Figure 7). Only INPUT and the positive control showed the predicted band using human RegIV primer-A-C, G but not in GLI-Ab, IgG, and negative groups (data not shown). The results of sequence analysis showed that the sequences were the same as that of the RegIV gene promoter of site 4 (Figure S5, S6, S7). All data suggested that GLI1 was bound to the RegIV gene promoter of site 4 (GATCATCCA), and regulated RegIV in PC through the HH signaling pathway.

**Figure 7:** Modulation of GLI1 binding on RegIV promoter was assessed by Chromatin immunoprecipitation (ChIP) assay. The locations of RegIV primer-A-G in the promoter region of RegIV gene. The numbers on the schematic of the RegIV gene (numbers 1–5) correspond to the potential GLI1 binding sites. P represents the transcriptional start site. Lysates from PANC-1 cells were subjected to Chromatin immunoprecipitation by anti-GLI1 antibody. Human RegIV primer-A-G were used to amplify the RegIV promoter region containing the putative GLI1-binding site. Sonicated chromatin were used as INPUT DNA control. IgG, RNA polymerase II, and β-actin Ab were used as random controls, positive controls, and negative controls. (B) Only INPUT, positive control, and GLI1-Ab showed the predicted band in ethidium bromide-stained agarose gels using the CHIP-PCR products which were amplified by RegIV primer-D(i), RegIV primer-E(ii), and RegIV primer-F(iii). No detectable transcript was observed in amplified template from IgG or negative control and a positive control lane confirmed the expected fragment. Molecular weight standards (Marker) were used to estimate the size of the amplified bands.

### Confirmation of GLI1 bound to the RegIV promoter by EMSA

As described above, the GLI1 binding site in the promoter region of the RegIV gene was confirmed with ChIP-PCR. We then used EMSA assays to directly address whether GLI1 binds RegIV *in vivo*. We synthesized specific oligonucleotides containing the GLI1 element present in the RegIV promoter in EMSA experiments with nuclear extracts from PANC-1 cell lines. As shown in Figure 8, incubation of PANC-1 cells extracts with the biotin-labeled GLI1-RegIV sequence produced a DNA-protein band shift. These DNA-protein complexes were specific to the GLI1 site by successful competition assays using different folds of excess unlabeled GLI1-RegIV and mutant labeled GLI1-RegIV oligonucleotides. To confirm the binding of GLI1 to the GLI1-RegIV sequence, these EMSA reactions were further incubated with anti-GLI1 antibody. As shown in Figure 8, the addition of this antibody resulted in a supershifted complex in addition to the DNA-protein band. These data demonstrated the presence of GLI1 in the nuclear protein complex that binds the GLI1 binding site of the RegIV promoter (−528∼−520).

**Figure 8:** Analyses of the binding of GLI1 to the Reg IV promoter by Electrophoretic Mobility Shift Assays (EMSA). EMSA was performed with nuclear extracts of PANC-1 cells (lanes 2 to 7) or without nuclear extracts (lane 1). The RegIV probe was generated by annealing single-stranded and end-labeled oligonucleotides containing the RegIV promoter region (nucleotides −528∼−520). Competition experiments were performed using 1-fold (lanes 3), 10-fold (lanes 4), and 100-fold (lanes 5) excess of unlabeled oligonucleotides, respectively (lanes 3 to 5) or 100-fold mutant labeled oligonucleotides (lane 6). For super-shift, anti-GLI1 antibody (lane 7) was incubated with nuclear extracts before being added to the reaction.

## Discussion

In this study, we confirmed that GLI1 and RegIV were overexpressed in PC tissue and cell lines, confirmed by other reports [12], [20], [32]. We also demonstrated a significantly positive correlation between the expression of GLI1 and RegIV. RNA interference and overexpression experiments showed that RegIV expression changed with GLI1 expression in PC cell lines; this was confirmed by CHIP and EMSA. This is the first report that GLI1 can modulate RegIV expression by binding to the RegIV gene promoter, and that GLI1 is a RegIV transcriptional factor.

The HH signaling pathway, including transcription factor GLI1, is involved in the development of many kinds of cancers, including PC [12], [13], [32]–[35]; however, the mechanism has not been fully elucidated. Thus far, only a few downstream targets of GLI1 have been identified, including GLI1, PTCH, HHIP, CCND, Snail, Bcl-2, cyclin D2, FOX-F1, -L1, -M1, Follistatin, and N-Myc [36]. We demonstrated that the HH-GLI1 signaling pathway could regulate RegIV expression by a serie of experiments, including CHIP and EMSA. In our literature review, we learned that RegIV expression in different cell types was associated with regeneration, and cell growth, survival, adhesion, and resistance to apoptosis. RegIV is systematically overexpressed in stomach [24], colon [25], [26], and pancreas cancers [27], [28] and in diseases that predispose to colon cancer such as ulcerative colitis [29]. IHC analysis has confirmed RegIV expression in gastric, colorectal, and pancreatic carcinoma [27], [37], [38], and that RegIV has a potential role in diagnosing digestive tract neuroendocrine tumors [39]. RegIV gene amplification is an early event in pancreatic cancer development [30], and elevated RegIV was found in the sera of patients with PC [28]. PC-derived cells overexpressing RegIV protein grew more rapidly and were more resistant to gemcitabine treatment [30]. RegIV overexpression was thought to be associated with an unfavorable response to adjuvant chemoradiotherapy in patients with PC [40]. Other studies showed that RegIV was associated with a relatively favorable prognosis in patients with gallbladder carcinoma after surgical resection [41]. Thus, we concluded that the HH/GLI1/RegIV cascade may be an important pathway in PC development.

Chromatin immunoprecipitation (CHIP) is a reliable procedure used to determine whether a protein binds to or is localized to a specific DNA sequence *in vivo*. Through CHIP and promoter analysis, we identified a direct transcriptional target gene of GLI1, although the GLI1-binding element (GATCATCCA) showed a 2 nucleotide difference (underlined) from a previously identified 9-nucleotide GLI1-binding sequence (GACCACCCA) [42]. EMSA is one of the most sensitive methods for studyting protein-DNA interactions. This procedure can determine if a protein or mixture of proteins is capable of binding to a given DNA sequence. “Supershift assay” is a term used to unambiguously identify a protein present in the protein-nucleic acid complex. The EMSA and supershift assay also confirmed GLI1 to be bound on site 4 of the RegIV promoter motif. Those results suggested that GLI1 can bind to RegIV gene promoters on site 4 *in vivo*. Based on these results, we concluded that GLI1 transcriptionally regulates RegIV gene in PC cells.

Although the biological function of RegIV is poorly understood, it has been reported that RegIV may function as a growth and antiapoptotic factor in gastric, colon, and pancreatic cancers [27], [29], [43], [44]. The expression of RegIV may contribute to liver metastasis through induction of MMP7 by RegIV [44], and is a potent activator of the EGFR/Akt/AP-1 signaling pathway in colon cancer cells. It also increases the expression of Bcl-2, Bcl-xl, and survival proteins, all associated with the inhibition of apoptosis [44]. However, the role of RegIV in migration and invasion, and whether GLI1 contributes to proliferation, migration, and invasiveness through RegIV regulation in PC is still unclear. Whether RegIV is transcriptionally regulated by GLI1, thus imposing its effect on pancreatic carcinogenesis, the pathways responsible require further investigation. The coherence of different molecular events would be partly elucidated by revealing the mechanism of transcriptional regulation between GLI1 and RegIV, which may be determined by investigating the effects of GLI1 and RegIV on common signaling pathways such as the EGFR/Akt/AP1 cascade, as reported recently both in HH and RegIV. Our work may contribute to the body of research on pancreas carcinogenesis and provide insight into the correlated network of signaling pathways through the GLI1/RegIV axis.

In conclusion, the SHH-GLI1 signaling pathway regulates the transcription of RegIV gene in PC. This is the first report that demontrates GLI1 as a transcriptional factor that regulates RegIV expression in PC. Our work may help to elucidate the molecular mechanism of the SHH-GLI1 signaling pathway and promote earlier diagnosis and treatment of PC. The newly identified GLI1/RegIV axis provides a new insight into PC pathogenesis. Additional studies are required to determine whether the biological behavior of GLI1 in PC may be achieved by regulating RegIV.

## Supporting Information

Figure S1 **The result of sequence analysis of positive clone products in overexpression-GLI1 lentiviral vector construction.** The resultant 3320-bp fragment was confirmed by sequencing which is same with the sequence of the GLI1 gene expression region in GenBank (NM_005269.2).
(TIF)

Figure S2 **Transduction efficiency of PANC-1 cells by lentivirus vector were evaluated by FCM.** Cells were transfected with GFP-vector. Transduction efficiency based on the fluorescent signalwas analyzed by FCM. (A) PANC-1 cells without transfection were used as the blank control; (B) Cells transfected with GFP-shRNA as random control; (C) Cells transfected with GLI1-shRNA as experiment group.
(TIF)

Figure S3 **Transduction efficiency of PANC-1 cells by lentivirus vector, phase contrast and GFP expression under a fluorescent microscope.** Transduction efficiency of PANC-1 cells by GLI1 silencing vector. PANC-1 cells were transfeced with the GLI1-shRNA vector. The corresponding phase-contrast image(left panel), the GFP fluorescence (middle panel) and the merged image (right panel) are shown at a magnification of ×200. GFP expression reveals high transduction efficiency, with more than 90% of cells being transduced.
(TIF)

Figure S4 **Electropheretogram of sonicated chromatin solution in different conditions.** Sonicated chromatin solution in different conditions were electrophoresed on 1.5% agarose gel containing ethidium bromied. DNA sizes appear smear at a range of 100 bp to 1 kb range in 80 W group.
(TIF)

Figure S5 **The result of sequence analysis of CHIP products which amplified by RegIV primer-D.** The result showed that the sequence amplified with RegIV primer-D is the same as that of RegIV gene promoter region containing GLI1-binding site 4.
(TIF)

Figure S6 **The result of sequence analysis of CHIP products which amplified by RegIV primer-E.** The result showed that the sequence amplified with RegIV primer-E is the same as that of RegIV gene promoter region containing GLI1-binding site 4.
(TIF)

Figure S7 **The result of sequence analysis of CHIP products which amplified by RegIV primer-F.** The result showed that the sequence amplified with RegIV primer-F is the same as that of RegIV gene promoter region containing GLI1-binding site 4.
(TIF)
